# Application of CT Imaging in Differential Diagnosis and Nursing of Endocrine Tumors

**DOI:** 10.1155/2022/4071081

**Published:** 2022-08-08

**Authors:** Xue Jiang, Weiwei Xu, Ying Zhao

**Affiliations:** ^1^Department of Endocrinology, The Second Hospital of Jilin University, Changchun, Jinlin 130000, China; ^2^Department of Oncology and Hematology, The Second Hospital of Jilin University, Changchun 130000, China

## Abstract

In order to investigate the value of preoperative X-ray computed tomography (CT) in predicting the pathological grade of pancreatic neuroendocrine tumors. This paper retrospectively analyzed the CT image examination of pancreatic neuroendocrine tumors, the image characteristics of G-NEC detected by CT image, and the detection of GST by spiral CT. In order to clearly diagnose and evaluate the size and scope of the focus, whether there is adjacent tissue invasion, metastasis, and treatment effect, CT, MR, PET-CT, nuclide specific imaging, and other imaging methods are widely used in the medical treatment of pNEN patients. These imaging methods have the advantages of noninvasive, rapid imaging, objective image medium, and strong repeatability. If the pathological grade of pNEN patients can be obtained by imaging examination before operation, it will be of great benefit to the formulation of treatment strategies and the prediction of clinical outcomes. Combining CT image performance with imaging omics characteristics to establish a prediction model that can develop a better auxiliary decision-making tool for clinical practice. Different pathological grades prompt clinicians to provide personalized and accurate medical treatment for patients, and reduce excessive medical treatment or wrong judgment caused by unclear preoperative diagnostic information.

## 1. Introduction

Pancreatic ductal adenocarcinoma (PDAC) is the most common malignant tumor of the pancreas, accounting for about 80% of pancreatic tumors. It is a tumor with little blood supply. Its clinical and imaging manifestations need to be differentiated from pancreatic neuroendocrine tumor (PNET) and solid pseudopapilloma of the pancreas (SPTP) [1]. Although PNET is a tumor with rich blood supply, there is no obvious enhancement after about 41%∼49% enhancement. SPTP has malignant potential. The focus is mainly composed of solid components and is small, which is difficult to distinguish from PDAC and PNET. The imaging findings of PDAC, SPTP, and PNET overlap, and there are some difficulties in preoperative differential diagnosis. Based on image pixel intensity and spatial distribution, texture analysis can reflect tumor heterogeneity. Clinical features of supratentorial PNET in adults are not specific, but the tumor is often large, which can cause intracranial hypertension and space-occupying symptoms and signs. Patients have increased intracranial pressure symptoms as the first symptoms, such as headache and vomiting. In this group, there were 5 patients with symptoms of intracranial hypertension such as headache and vomiting, and 3 patients with a simple headache. However, there is little research on texture analysis related to pancreatic tumors.  Figure 1 shows the types of pancreatic tumors.

## 2. Literature Review

To address this research question, Niu et al. analyzed the relationship between CT texture features and PNET differentiation grade, and found that CT texture features were better than traditional CT image features in evaluating PNET differentiation grade [2]. Emori et al. quantitatively analyzed the correlation between CT texture features and the overall survival rate of PDAC, and found that texture features (heterogeneity and inverse gap) may become a biomarker for preoperative assessment of the overall survival rate of PDAC [3]. Chen et al. used a single texture feature to have a good or very good diagnostic efficiency in differentiating pancreatic tumors, indicating that texture features can distinguish subtle differences between different types of pancreatic tumors [4]. Zhang et al. analyzed and compared the clinical diagnostic value of CT in 21 cases of G-NEC and 34 cases of GST by collecting the imaging, clinical, and pathological data [5]. Wei et al. retrospectively analyzed the clinical and CT findings of 7 cases of colon NEN to improve the understanding of the disease [6]. Winter et al. studied that 4 of the 7 patients had distant metastasis at the time of visit, including 2 cases of multiple liver metastasis, 2 cases of ovarian, peritoneal omental, and mesangial metastasis, and 1 case of ovarian metastasis complicated with renal sinus and retroperitoneal lymph node metastasis. The patient's condition progressed rapidly. Four patients had new retroperitoneal lymph node, lung, lumbar vertebra, and liver metastasis after 2 months of re-examination, and one patient had liver metastasis after half a month of re-examination [7]. Li et al. believe that GST is a mesenchymal tumor of the stomach, which has multiple differentiation potentials. It is more common in people over 40 years old and more common in women than men. Gastrointestinal bleeding is the most common symptom of GST, which is mostly caused by tumor necrosis or mucosal ulcer. Therefore, it also shows uneven enhancement under CT enhancement, as shown in Figure 2. Tumor whole-body tomography: lung cancer screening [8].

## 3. Analysis

### 3.1. CT Examination Method Analysis

A GE LightSpeed 64 row spiral CT scanner is adopted. Scanning parameters are as follows: tube voltage 120 kV, tube current 200∼250 m As, scanning layer thickness 5 mm, and layer spacing 5 mm. Place the injection syringe vertically upward, the A-tube syringe uses a disposable aspiration tube to aspirate the contrast agent (ordinary enhanced ioversol or vascular CTA iodine), and the B-tube syringe uses a plastic needle to aspirate. Inhale an appropriate dose of 0.9% normal saline and strictly follow the aseptic technique when drawing medicine. After fasting for 8 h before CT examination, all patients were scanned in the supine position, ranging from the top of the diaphragm to both the kidneys to the lower pole. After a plain scan, 1.5 ml/kg of a contrast agent (ornamac) was injected through the median elbow vein. As an auxiliary equipment in the radiology diagnosis and treatment system, the high-pressure injector is gradually applied clinically with the development of X-ray, rapid film changer, image intensifier, and artificial contrast agent. The basic function of the high-pressure syringe is to inject a sufficient amount of a high-concentration X-ray contrast agent into the examination site quickly and accurately through percutaneous puncture into the blood vessel or through the original orifice of the human body within a certain period of time, which can diagnose the lesion. Angiography and treatment. were conducted with a high-pressure syringe at a rate of 3.5ml/s. Three-phase dynamic enhanced images of the arterial phase, venous phase, and delayed phase were collected at intervals of 30 s, 60 s, and 180 s respectively.

#### 3.1.1. Imaging signs

CT imaging signs were analyzed by 2 radiologists (with more than 10 years of experience) with rich experience in abdominal imaging diagnosis, and consistent diagnostic results were obtained through discussion [9]. Read the patient's CT image in the hospital image archiving and communication system (PACS), and analyze the patient's image features, including the following: tumor location: pancreatic head and neck (including uncinate process), pancreatic body, pancreatic tail, or multiple parts in the pancreas. Size: expressed by the maximum diameter line of the tumor measured in the cross section, and the unit is em. Plain scanning density: low, equal, and high density. Calcification: whether there is calcification during the plain scan. Texture: according to the proportion of cystic and solid components, it can be divided into solid type, cystic and solid type, and cystic type. Boundary: clear boundary (smooth tumor edge) or unclear boundary (rough tumor edge or infiltration). The enhancement method: uniform and uneven. Peak enhancement intensity period: the CT value of the lesion was measured in each period of enhancement, and the maximum period was determined. Pancreatic duct dilatation refers to the widening of the pancreatic duct due to some reasons. When doing some imaging tests such as CT or MRI, it is often found. It is caused mainly because of the following reasons: first, the common bile duct or when there are stones in the pancreatic duct, it may cause the pancreatic duct to dilate, usually with abdominal pain, jaundice, fever, and other symptoms. Second, when there are benign and malignant lesions in the common bile duct, duodenum, or pancreas, such as benign and malignant tumors, inflammation, and parasites, the pancreatic duct can be significantly dilated, especially malignant tumors, which are often accompanied by tumor markers. Pancreatic duct dilatation: measure the widest part of the pancreatic duct; if the diameter exceeds 0.35 cm, it is defined as pancreatic duct dilatation. Bile duct dilatation: measure the widest part of the common bile duct at the upper edge of the pancreas; if the diameter is greater than 0.9 cm, it is defined as dilatation. Vascular invasion: the invasion of the common hepatic artery, splenic artery and vein, gastroduodenal artery, superior mesenteric artery and vein, and portal vein were observed. The criteria of invasion were vascular occlusion, stenosis, or more than half of the circumference in contact with the tumor. Peripheral organ invasion: whether it invades the spleen, duodenum, and stomach. Distant metastasis: liver, bone, lung, or lymphatic metastasis [10, 11].

#### 3.1.2. Imageomics

Feature extraction CT images were sketched by 2 radiologists with rich experience in abdominal image diagnosis, and consistent diagnostic results were obtained through discussion. DICOM images of abdominal enhanced CT in the arterial and venous phase were obtained from the hospital image archiving and communication system (PACS), and all original CT images were normalized. The region of interest (ROI) of the CT images in the arterial phase and venous phase are automatically segmented in ITK-SNAP by using the computer automatic segmentation algorithm, avoiding the pancreatic parenchyma, duodenum, and blood vessels around the tumor, and then, the automatically segmented images are manually adjusted layer by layer. Finally, the multilevel ROI is automatically fused into the volume of interest (VOI) [12]. The segmented image was guided by using the PyRadiomics software to standardize the intensity of ROI region and extract radiomics features. Hemangioma is a common benign tumor, including arterial hemangioma and venous hemangioma. There are two kinds of blood vessels in the human body, one is an artery and the other is a vein. The tumor VOI of the arterial phase and venous phase of each patient's CT image obtained image omics features, including gray histogram, shape feature (3D), and texture features, based on gray level co-occurrence matrix, gray level size region matrix, gray level run length matrix, adjacent gray level tone difference matrix, and gray level dependence matrix.

### 3.2. CT Imaging of Pancreatic Neuroendocrine Tumors

The incidence rate of pancreatic neuroendocrine tumors (PNENs) is low, accounting for only 1%∼3% of all pancreatic tumors, but the incidence rate and prevalence have increased in recent years. According to the general classification framework of neuroendocrine tumors proposed by the international agency for research on cancer - World Health Organization (IARCWHO), PNENs are divided into well-differentiated pancreatic neuroendocrine tumors (PanNETs) and poorly differentiated pancreatic neuroendocrine carcinoma (PanNECs). PanNETs were divided into three grades (G1, G2, and G3) according to the mitotic number and the Ki-67 index. The choice of treatment methods for PNENs mostly depends on the pathological grade of the tumor, and the choice of surgery and surgical methods depend on the size, location, and histopathological grade of the tumor [13]. At present, a large number of studies have proved that the grading system of pancreatic neuroendocrine tumors has a great correlation with their prognosis. The 5-year survival rates of G1, G2, and G3 PanNETs are 75%, 62%, and 7%, respectively. Pancreatic neuroendocrine tumors (PanNETs) are relatively rare tumors whose incidence has increased in recent years. Functional PanNETs are detected early now due to symptoms and associated complications, whereas nonfunctional PanNETs (NF-PanNETs) often persist for many years. Therefore, accurately predicting the grading of PanNETs before operation is of great significance to the selection of clinical treatment schemes and the evaluation of late prognosis. CT imaging is the main imaging method for pancreatic tumor localization, TNM staging, and monitoring treatment response. However, CT examination lacks imaging signs for pathological grading. At present, endoscopic ultrasound-guided fine-needle aspiration (EUS-FNA) is a more accurate method to obtain the pathological grade of pNEN before operation. Endoscopic ultrasound-guided fine-needle aspiration cytology (EUS-FNA) is to puncture a fine needle through an endoscopic biopsy channel into the target tissue under the guidance of endoscopic ultrasound to obtain the target cells and tissues for pathology and diagnosis. However, EUS-FNA is an invasive method. In many cases, the volume of tissue obtained by aspiration is limited and it is difficult to reflect the heterogeneity of the tumor, because the depth of the pancreas is unable to obtain the tumor tissue. Imageomics is a new research field of high-throughput extraction of medical image features. By extracting, analyzing, and predicting the image features of the region of interest related to the target, and combining with clinical pathological data and image signs, it develops personalized tools to assist clinical decision-making or predict clinical endpoint events. At present, imageomics has been applied to the prognosis evaluation of pancreatic diseases and differential diagnosis of benign and malignant tumors. Some studies show that imageomics has potential prospects in predicting the pathological grade of pancreatic neuroendocrine tumors [14, 15].

### 3.3. CT Image Detection G-NEC Image Features

G-NEC is relatively rare. It originates from the midgut chromaffin cells of the precarboxylation system of the digestive tract and has the function of secreting bioactive peptides, hormones, and neurotransmitters. However, in recent years, its incidence rate has shown an upward trend, and it is more common in men, with a male to female ratio of about 3 : 14. The clinical manifestations of G-NEC are mostly gastrointestinal symptoms such as abdominal distension, abdominal pain, and black stool, and few cases are typical symptoms such as skin flushing, organ spasm, asthma, and diarrhea. G-NEC is highly malignant, invasive, and prone to lymph node metastasis. Surgical treatment is usually performed according to the principle of gastric adenocarcinoma surgery, but adjuvant chemotherapy is recommended if it enters the T4 stage. Retrospective analysis of the data showed that the CT image features of G-NEC were mainly as follows: most of them occurred under the cardia and the gastric body, most of them were single and prone to lymph node metastasis, most of the tumors were irregular and had thickened gastric wall, and most of the enhanced CT showed uneven and obvious enhancement. Most cases were further enhanced in the venous phase, which confirmed that G-NEC had delayed enhancement and was mostly rich in blood supply, which was consistent with previous reports. However, previous literature has shown that most of the G-NEC showed uniform enhancement. At present, the diagnosis of G-NEC mainly depends on pathological examination, especially immunohistochemistry. CgA, neuron specific enolase (NSE), and syn are the most widely used. CgA and syn have high specificity and NSE sensitivity. Some scholars have found that CGA is related to tumor development and prognosis, so it can be used as a marker to detect tumor recurrence and evaluate prognosis [16, 17].

### 3.4. GST Detection by Spiral CT

GST is a mesenchymal tumor imprint that occurs in the stomach. It has multiple differentiation potentials. It is more common in people over 40 years of age than in women. Gastrointestinal bleeding is the most common symptom of GST. It is mostly caused by tumor necrosis or mucosal ulcer. Therefore, it also shows uneven intensification under CT enhancement. GST has a potential malignant tendency. Early detection is of great significance to ensure the life safety of patients. Imaging examination is currently the main detection method of GST, of which spiral CT is the most widely used [18]. Most of GST had clear and smooth edges and abundant blood supply on CT. The tumors in the arterial phase showed mild or moderate enhancement, while those in the portal vein phase showed delayed enhancement. GST can be divided into intragastric type (the tumor is located under the mucosa and grows into the lumen), extragastric type (the tumor is located under the gastric serosa and grows into the lumen) (C1994-2020 China Academic Journal ETlectronic Pu), and mixed type according to the tumor growth mode. GST has abundant blood supply, most of which are hematogenous metastasis or intraperitoneal implant metastasis; lymph node metastasis and liver metastasis are rare [19, 20]. GST most often occurs in the gastric body. Most of them are round-like masses with clear boundaries, showing expansive growth. The research of GST mainly focuses on the judgment of benign and malignant. The pathological judgment of benign and malignant is mostly based on the size and mitotic rate of the tumor: when the tumor diameter is less than 5.0 cm and the tumor shows homogeneous enhancement, it is mostly benign; when the diameter ≥5.0 cm and combined with cystic degeneration, necrosis and hemorrhage of different degrees, uneven enhancement under CT enhancement, the possibility of malignancy is greater [21]; benign GST mitotic images were rare; the density and cell atypia of malignant GST cells increased, and the mitotic images were ≥10/50 high power fields (HPF). In addition, the marginal contour of the mass, the presence or absence of migrating vessels in the tumor, the clear boundary between the tumor and the surrounding tissues, and the invasion and metastasis of the surrounding organs are of great significance for the judgment of benign and malignant tumors. The most characteristic immune markers of GST are CD34 and CD117, of which CD117 is the most prominent. The 5-year relapse-free survival rate of GST after simple surgical resection can reach 70.5%. Therefore, early detection and treatment are of great significance [22].

### 3.5. Discussion

Early and accurate pathological grading is of great significance to the choice of treatment and the analysis of prognosis. At present, the acquisition of clinical pathological specimens mainly depends on surgical resection specimens and endoscopic guided fine-needle biopsy (EUS _FNA). Although EUS-FNA can obtain tissue samples before surgery, the tissue samples obtained by the puncture are limited, which may produce a false negative phenomenon or underestimate the tumor grade, and sample processing and sampling errors may also lead to misjudgment of tumor invasiveness; in addition, EUS-FNA is an invasive examination, and the sampling level is related to the level of the operator to some extent, so it is sometimes difficult to obtain pancreatic tail samples [23].

In order to clearly diagnose and evaluate the size and scope of the focus, whether there is adjacent tissue invasion, metastasis and treatment effect, CT, MR, PET-CT, nuclide specific imaging, and other imaging methods are widely used in the medical treatment of pNEN patients. These imaging methods have the advantages of noninvasive, rapid imaging, objective image medium, and strong repeatability. If the pathological grade of pNEN patients can be obtained by imaging examination before operation, it will be of great benefit to the formulation of treatment strategies and the prediction of clinical outcomes. Scholars at home and abroad have carried out many studies in this direction and found that tumor size >2 cm, relatively solid, irregular shape, unclear boundary, low enhancement in the arterial phase, low apparent diffusion coefficient (ADC) value, as well as signs associated with dilation of main pancreatic duct, vascular invasion, lymphadenopathy, organ metastasis, etc., are related to a higher pathological grade and poor prognosis. However, most of the existing research results are based on small samples and single center research. The diagnostic efficacy of the research is not ideal, and there is a lack of external verification, so the clinical application value is limited [24]. The comprehensive model combines the tumor boundary, surrounding organ invasion, and multifactor analysis of meaningful imaging omics characteristics of image performance, and its prediction efficiency is better than the image performance model and the imaging omics model, showing that the comprehensive model has a stronger ability to predict the pathological grade of PanNETs [25]. By combining CT image performance with imaging omics characteristics to establish a prediction model, we can develop a better auxiliary decision-making tool for clinical practice. Different pathological grades prompt clinicians to provide personalized and accurate medical treatment for patients and reduce excessive medical treatment or wrong judgment caused by unclear preoperative diagnostic information.

## 4. Conclusion

The retrospective analysis of this paper shows that imagemics is a new research field of high-throughput extraction of medical image features. By extracting and analyzing the image features of the region of interest related to the prediction target, and combining with clinical pathological data and image signs, we can develop personalized tools to assist clinical decision-making or predict clinical endpoint events. At present, imaging omics has been applied to the prognosis evaluation of pancreatic diseases and differential diagnosis of benign and malignant tumors. Some studies show that imaging omics has potential prospects in predicting the pathological grading of pancreatic neuroendocrine tumors.

## Figures and Tables

**Figure 1:** Types of pancreatic tumors.

**Figure 2:** Tumor whole-body tomography imaging: lung cancer screening.

## Data Availability

The data used to support the findings of this study are available from the corresponding author upon request.

## References

[1] Zheng X. Z., Ma J. H., Chen T. B. (2020). Application of molecular analysis in differential diagnosis of ovarian adult granulosa cell tumors. *Chinese Journal of Pathology*.

[2] Niu S., Huang J., Li J. (2020). Application of ultrasound artificial intelligence in the differential diagnosis between benign and malignant breast lesions of bi-rads 4a. *BMC Cancer*.

[3] Emori M., Takashima H., Iba K. (2021). Differential diagnosis of fibroma of tendon sheath and giant cell tumor of tendon sheath in the finger using signal intensity on t2 magnetic resonance imaging. *Acta Radiologica*.

[4] Chen P., Dong B., Zhang C., Tao X., Wang P., Zhu L. (2020). The histogram analysis of apparent diffusion coefficient in differential diagnosis of parotid tumor. *Dentomaxillofacial Radiology*.

[5] Zhang Z. C., Hu J., Kong Y. Y., Ren M., Cai X. (2021). Application of immunohistochemical staining of bcl-2, ber-ep4, cd10, ck20, and ki-67 in differential diagnosis between trichoblastoma and basal cell carcinoma. *Zhonghua bing li xue za zhi Chinese journal of pathology*.

[6] Wei J., Zhu R., Zhang H., Li P., Okasha A., Muttar A. K. (2021). Application of pet/ct image under convolutional neural network model in postoperative pneumonia virus infection monitoring of patients with non-small cell lung cancer. *Results in Physics*.

[7] Winter J. M., Sheehan-Hennessy L., Pedersen S. K., Wassie M. M., Young G. P., Symonds E. L. (2021). Application of a colorectal cancer ctdna methylation test in endocrine cancers. *Journal of Clinical Oncology*.

[8] Li X., Nie P., Zhang J., Hou F., Ma Q., Cui J. (2022). Differential diagnosis of renal oncocytoma and chromophobe renal cell carcinoma using ct features: a central scar-matched retrospective study. *Acta Radiologica*.

[9] Wei W., Huang X., Zeng L., Zhong J. (2022). Application of psychological elastic development model in postoperative trauma growth of patients with esophageal cancer. *Journal of Cancer Therapy*.

[10] Yue X., Zhong L., Wang Y. (2022). Value of assessment of different neoplasias in the adnexa in the differential diagnosis of malignant ovarian tumor and benign ovarian tumor: a meta-analysis. *Ultrasound in Medicine and Biology*.

[11] Shi X., Du T., Zhu D. (2021). High-dose dexamethasone suppression test is inferior to pituitary dynamic enhanced MRI in the differential diagnosis of ACTH-dependent Cushing’s syndrome. *Endocrine*.

[12] Vernuccio F., Porrello G., Cannella R. (2021). Benign and malignant mimickers of infiltrative hepatocellular carcinoma: tips and tricks for differential diagnosis on ct and mri. *Clinical Imaging*.

[13] Panigrahi C., Jha S., Kumar P., Mishra T. S., Sasmal P. K., Adhya A. K. (2022). Squamous metaplasia in a borderline phyllodes tumor—an undocumented histological finding in male breast: report of a case and review of literature. *International Journal of Surgical Pathology*.

[14] Zhao Y., Lin S., Wu J., Lai J., Li L. (2021). A study of the clinical application value of ultrasound and electrocardiogram in the differential diagnosis of cardiomyopathy. *American Journal of Tourism Research*.

[15] Shi J., Liu X., Ming Z. (2021). Value of combined detection of cytokines and tumor markers in the differential diagnosis of benign and malignant solitary pulmonary nodules. *Zhongguo fei ai za zhi = Chinese journal of lung cancer*.

[16] Yang Z., Gong Y., Ji M., Yang B., Qiao Z. (2020). Differential diagnosis of pancreatoblastoma (pb) and solid pseudopapillary neoplasms (spns) in children by ct and mr imaging. *European Radiology*.

[17] Luo X., Preciado C., Nayak A. (2022). Renal oncocytoma with both lymphovascular invasion and prominent intracytoplasmic vacuole-like spaces: a case report and review of the literature. *International Journal of Surgical Pathology*.

[18] Ratasvuori M., Sormaala M., Kinnunen A., Lindfors N. (2022). Ultrasonography for the diagnosis of carpal tunnel syndrome: correlation of clinical symptoms, cross-sectional areas and electroneuromyography. *Journal of Hand Surgery*.

[19] Liu R., Guo Z., Huang J., Li J., Tan Q., Luo Q. (2022). Identification of a 7-mirna signature for predicting the prognosis of patients with lung adenocarcinoma. *Experimental Biology and Medicine*.

[20] Ozsen M., Saraydaroglu O., Yirmibes S., Coskun H. H. (2022). Lesions that mimic malignant tumors in nasopharyngeal biopsies: case series of 10 years. *Tumori Journal*.

[21] Li G., Liu F., Sharma A. (2021). Research on the natural language recognition method based on cluster analysis using neural network. *Mathematical Problems in Engineering*.

[22] Selva D., Nagaraj B., Pelusi D., Arunkumar R., Nair A. (2021). Intelligent network intrusion prevention feature collection and classification algorithms. *Algorithms*.

[23] Liu X., Ma C., Yang C. (2015). Power station flue gas desulfurization system based on automatic online monitoring platform. *Journal of Digital Information Management*.

[24] Huang R., Zhang S., Zhang W., Yang X. (2021). Progress of zinc oxide-based nanocomposites in the textile industry. *IET Collaborative Intelligent Manufacturing*.

[25] Kaabar M. K. A., Kalvandi V., Eghbali N., Samei M. E., Siri Z., Martínez F. (2021). A generalized ML-hyers-ulam stability of quadratic fractional integral equation. *Nonlinear Engineering*.

